The article "TRIM66 Promotes Malignant Progression of Non-Small-Cell Lung Cancer Cells via Targeting MMP9" was published in 2022. Journal: Comput Math Methods Med.

# TRIM66 Promotes Malignant Progression of Non-Small-Cell Lung Cancer Cells via Targeting MMP9

**DOI:** 10.1155/2022/6058720

**Published:** 2022-07-21

**Authors:** Yufen Xu, Qi Yang, Zhixian Fang, Xiaoli Tan, Ming Zhang, Wenyu Chen

**Affiliations:** ^1^Department of Oncology, Affiliated Hospital of Jiaxing University, No. 1882, Zhonghuan South Road, Nanhu District, Jiaxing, Zhejiang Province 314001, China; ^2^Department of Respiratory Medicine, Affiliated Hospital of Jiaxing University, Jiaxing, Zhejiang Province 314001, China

## Abstract

Lung cancer has a higher incidence and mortality rate than other cancers, and over 80% of lung cancer cases were classified as non-small-cell lung cancer (NSCLC). TRIM66 is one of the crucial members of TRIM, which has a deep connection with the behavior of various malignant tumors. But it remains uncertain regarding its exact function and underlying mechanism in NSCLC. In our study, qRT-PCR and Western blot were employed to validate that TRIM66 was overexpressed in NSCLC. The migration, invasion, and epithelial-mesenchymal transformation (EMT) progression of NSCLC cells were determined by Western blotting and Transwell experiments after knocking down TRIM66, and it was found that knockdown TRIM66 inhibited the migration, invasion, and EMT processes of NSCLC cells. Next, the binding relationship between TRIM66 and MMP9 was verified by Co-IP assay. After determining the interaction between them, rescue assays showed that overexpression of MMP9 was capable to promote the migration, invasion, and EMT of NSCLC cells. However, the transfection of si-TRIM66 could reverse this facilitating effectiveness. To sum up, we concluded that by targeting MMP9, TRIM66 could exert a cancer-promoting role in the progression of NSCLC cells.

## 1. Introduction

The global cancer statistics indicated that the number of lung cancer diagnoses was about 1.8 million each year, which accounts for 13% of all newly diagnosed cancer cases [1]. Non-small-cell lung cancer (NSCLC) and SCLC are two subtypes of lung cancer [2]. NSCLC accounts for more than 80% of lung cancer cases [3]. And most patients present with advanced NSCLC at diagnosis. Though recent years have witnessed lots of improvement in early diagnosis and treatment of lung cancer, most of the treatment for NSCLC is surgery, chemotherapy, and radiation therapy [4]; the 5-year survival rate of NSCLC patients does not exceed 20% [3]. However, the genes associated with NSCLC and potential therapeutic targets are unclear. Hence, the current research focuses on identifying effective prognostic markers and possible therapeutic targets in NSCLC.

The tripartite motif-containing protein (TRIM) family participates in innate immunity to viruses, cell cycle, apoptosis, and so on [5, 6]. As one of the members, TRIM66 takes a part in the behavior of various cancers [7]. Existing studies indicate that the abnormal expression of TRIM66 in NSCLC can promote lymphatic and distant metastasis, which is a negative factor affecting prognosis [8]. Epithelial-mesenchymal transition (EMT) is an essential part of tumorigenesis as well as metastasis [8, 9]. The loss of E-cadherin and the increase in migratory and invasive behaviors and elevated levels of vimentin and N-cadherin are the features of EMT [10]. He et al. [11] found that the knockdown of TRIM66 can inhibit the EMT process. However, it remains unclear about the role of TRIM66 in NSCLC progression. And the enzymes that regulate the role of TRIM66 in NSCLC are not clear to us. Hence, research is needed.

The article "TRIM66 Promotes Malignant Progression of Non-Small-Cell Lung Cancer Cells via Targeting MMP9" was published in 2022. Journal: Comput Math Methods Med.

Matrix metalloproteinase 9 (MMP9) is a type IV collagenase that plays a crucial part in promoting cell migration and reepithelialization [12]. MMP9 is implicated with the malignant progression of cancer, including but not limited to invasion [13, 14], migration [15], metastasis [16], and angiogenesis [17]. On the basis of above findings, the speculation that MMP9 may be a potential biomarker and target has been investigated. However, how MMP9 works in NSCLC is rarely studied.

Our study focuses on TRIM66 by validating its expression level in NSCLC. Its targeted relationship in NSCLC with MMP9 was validated through ChIP experiment. Then, the migration, invasion, and epithelial-mesenchymal transformation (EMT) progression of NSCLC cells were determined by Western blotting and Transwell experiments after knocking down TRIM66. Our study can bring an improved comprehension of molecular mechanisms of NSCLC malignant progression and may provide potential targets for NSCLC.

## 2. Materials and Methods

### 2.1. Cell Culture

Human pulmonary alveolar epithelial cells (HPAEpiC) were procured from Shanghai Zhong Qiao Xin Zhou Biotechnology Co., Ltd, and NSCLC cell lines H460, H1299, and A549 were bought from Shanghai Cell Bank of the Chinese Academy of Sciences (Shanghai, China). Conditions for the cell culturing were as follows: alveolar epithelial cell culture medium for HPAEpiC, RPMI-1640 culture medium containing 10% high-quality fetal bovine serum (FBS) for H460 and H1299 (GIBCO, Art. No. 31800022, supplemented with 2.5 g/L glucose, 1.5 g/L NaHCO_3_, and 0.11 g/L sodium pyruvate, USA), and F12K medium containing 10% high-quality FBS for A549 (Sigma, Art. No. N3520, supplemented with 2.5 g/L NaHCO_3_, Germany). The culture conditions were 37°C and 5% CO_2_.

### 2.2. Plasmid Construction and Cell Transfection

siRNA of TRIM66 (si-TRIM66) and corresponding negative control (si-NC), overexpressed plasmid of MMP9 (oe-MMP9), and corresponding negative control (oe-NC) was designed by Sangon Biotech (Shanghai, China). All transfections were performed with Lipofectamine 2000 (Invitrogen, Carlsbad, CA, USA). Cells were collected 48 h after transfection.

The article "TRIM66 Promotes Malignant Progression of Non-Small-Cell Lung Cancer Cells via Targeting MMP9" was published in 2022. Journal: Comput Math Methods Med.

### 2.3. RNA Purification and qRT-PCR Analysis

RNA extraction was conducted complying strictly with the instructions of TRIzol (Life Technologies Corporation of Carlsbad, California, USA). Then, the RevertAid First Strand cDNA Synthesis Kit (Thermo Fisher Scientific, USA) was employed for the reverse transcription of RNA into cDNA. The SYBR Green PCR kit (Takara Bio, Otsu, Japan) was utilized for performing PCR amplification on a StepOne Real-Time PCR System (Thermo Fisher Scientific, USA). And the relative gene expression normalized by *β*-actin was calculated using the 2-^*ΔΔ*Ct^ method. The sequences of the PCR primers were as follows:

TRIM66 forward primer 5′-GCCCTCTGTGCTACTTACTCTC-3′, reverse primer 5′-GCTGGTTGTGGGGGTTACTCTC-3′

*β*-Actin forward primer 5′-CATGTACGTTGCTATCCAGGC-3′, reverse primer 5′-CTCCTTAATGTCACGCACGAT-3′

### 2.4. Western Blot

After lysing cells by lysis buffer, a bicinchoninic acid protein assay kit (Thermo Fisher Scientific, USA) was utilized for the measurement of protein concentration. Then, after electrophoresis in sodium dodecyl sulfate polyacrylamide gel electrophoresis (SDS-PAGE), proteins were transferred onto polyvinylidene difluoride membranes (Millipore, USA). Next, membranes were blocked with 5% skimmed milk. 2 h later, membranes were incubated with primary antibodies overnight at 4°C, which were then incubated with secondary antibody at room temperature for 1 h the next day. The membranes were finally developed following the electrochemiluminescence (ECL) kit (Pierce Biotechnology, USA). Western blot images were acquired using a ChemiDoc imaging system (Bio-Rad, USA). Antibody information is detailed in Table 1, and the internal reference used here was *β*-actin. Antibodies were all purchased from Invitrogen (Thermo Fisher Scientific, USA).

### 2.5. Transwell Assays

Transwell inserts (8 *μ*M pore size, Costar, Cambridge, MA, USA) were employed for the assessment of cell migration as well as invasion. 2 × 10^4^ cells were seeded in inserts without or precoated with Matrigel (BD, Franklin Lakes, USA) in the basolateral membrane using 200 *μ*l of FBS-free medium for migration or invasion analysis, respectively. 600 *μ*l of medium with 10% FBS was placed in the lower chamber. After incubation for 24 h at 37°C in 5% CO_2_, cells from the upper chamber that failed to migrate as well as invade were swabbed. Then, methanol was used for the cell fixing, 0.5% crystal violet for cell staining, and phosphate buffered saline (PBS) (Gibco; Thermo Fisher Scientific, Inc., USA) for cell washing. They were then photographed and counted under a microscope (Zeiss, Germany).

The article "TRIM66 Promotes Malignant Progression of Non-Small-Cell Lung Cancer Cells via Targeting MMP9" was published in 2022. Journal: Comput Math Methods Med.

### 2.6. Co-Immunoprecipitation (Co-IP) Assay

Cells were lysed for 30 min in Co-IP buffer supplemented with protease inhibitor mixture (Sigma-Aldrich, USA). The centrifugation of these lysates was conducted for 15 min at 12,000 rpm. The supernatant was then incubated with 20 *μ*l protein A/G beads (Santa Cruz, USA) for 30 min, followed by centrifugation at 1000*g* for 5 min at 4°C. Next, the immunoprecipitation of proteins lasted for more than 4 h by using TRIM66 antibody or control IgG antibody at 4°C. Protein A/G was added to capture antigen-antibody complexes. And through centrifugation, those agarose bead-antibody antigen complexes were collected and then washed three times using PBS. Next, they were eluted in boiling protein sample buffer under reducing conditions. In the end, proteins were separated by SDS-PAGE and analyzed by Western blot.

### 2.7. Statistical Analysis

SPSS 22.0 (IBM Corp., Armonk, NY, USA) and GraphPad Prism 6.0 software (GraphPad Inc., San Diego, CA, USA) were utilized for data analysis. All measured data were presented as mean ± SD. The comparison between the two groups was testified by *t*-test, and *p* < 0.05 indicated a significant difference.

## 3. Results

### 3.1. TRIM66 Is Highly Expressed in NSCLC Cells

TRIM66 expression in HPAEpiC, H460, H1299, and A549 was analyzed by Q-PCR, the result of which revealed a higher level of TRIM66 in NSCLC cells than that in human pulmonary alveolar cells (Figure 1(a)). The result of Western blot assay is consistent with the finding of Q-PCR (Figure 1(b)). These all displayed that TRIM66 was abnormally increased in NSCLC cells. In addition, we selected H1299 and A549 which enjoyed the highest expression for subsequent experiments.

### 3.2. TRIM66 Downregulation Restrains Invasion, Migration, and EMT Process of NSCLC Cells

Transfection of si-TRIM66 plasmid into NCI-H1299 cells and A549 cells was performed to assess the expression of TRIM66 and biological behaviors of TRIM66 in NSCLC cells. Here, TRIM66 expression was knocked down at first. And the transfection efficiency was examined using Q-PCR as well as Western blot (Figures 2(a) and 2(b)). Next, we conducted a Transwell assay for the detection of the effect that TRIM66 exerted on cell migration and invasion. Silencing TRIM66 did exert remarkable inhibiting effects on cell migration and invasion (Figures 2(c) and 2(d)). Then, we examined EMT-related proteins by Western blot, from the result of which we observed that the expression of N-cadherin, vimentin, and SNAIL was downregulated, and E-cadherin expression was upregulated in both cell lines. It was further demonstrated that the knockdown of siRNA-mediated TRIM66 restrained the EMT process (Figure 2(e)). Therefore, we suggested that knockdown of TRIM66 can restrain migration, invasion, and EMT process of NSCLC cells.

The article "TRIM66 Promotes Malignant Progression of Non-Small-Cell Lung Cancer Cells via Targeting MMP9" was published in 2022. Journal: Comput Math Methods Med.

### 3.3. The Bindings between TRIM66 and MMP2 or MMP9 Are Verified

MMP2 and MMP9 are considered to exert an important role in tumor metastasis [18]. To dig deeper into the regulatory mechanism that TRIM66 works in NSCLC cells, we tried to figure out the interactions between TRIM66, MMP2, and MMP9 by Western blot. Knockdown of TRIM66 could downregulate both MMP2 and MMP9 expression when compared to the control group (Figure 3(a)). Further, Co-IP was performed to investigate whether there was a physical binding between TRIM66 and MMP2 or MMP9, and the results revealed that Co-IP occurred only between TRIM66 and MMP9 (Figure 3(b)). Next, MMP9 level in NSCLC and pulmonary alveolar epithelial cells was also examined by Western blot, demonstrating that MMP9 was upregulated in NSCLC cell lines (Figure 3(c)). Based on the abovementioned findings, we could conclude that there was a direct interaction between TRIM66 and MMP9. And MMP9 displayed a high expression level in NSCLC cells.

### 3.4. TRIM66 Affects the Migration, Invasion, and EMT of NSCLC Cells by Mediating MMP9

To further verify the regulatory relationship between TRIM66 and MMP9 in NSCLC cells, we transfected si-NC + oe-NC, si-NC + oe-MMP9, and si-TRIM66 + oe-MMP9 into H1299 cells and A549 cells. Firstly, transfection efficiency testified by Western blot, illustrating that MMP9 displayed a remarkably upregulated expression in the si-NC + oe-MMP9 group relevant to the control group, but after simultaneous silencing TRIM66, the upregulation in MMP9 expression decreased (Figure 4(a)). Secondly, Transwell assay results demonstrated that enforced expression of MMP9 fostered migration and invasion of NCI-H1299 and A549 cells, while transfection of si-TRIM66 could reverse the promoting effect of oe-MMP9 (Figures 4(b) and 4(c)). Next, we found that compared with controls, overexpression of MMP9 only upregulated N-cadherin, vimentin, and SNAIL expression and downregulated E-cadherin expression relevant to the control group, which was conducive to EMT. However, simultaneous silencing of TRIM66 expression could revert these results compared with overexpression of MMP9 alone (Figure 4(d)). Thus, influence of overexpressed MMP9 on NSCLC cell migration, invasion, and EMT was reversed by silencing TRIM66.

The article "TRIM66 Promotes Malignant Progression of Non-Small-Cell Lung Cancer Cells via Targeting MMP9" was published in 2022. Journal: Comput Math Methods Med.

## 4. Discussion

In the past decade, a variety of oncogenes have been discovered, such as KRAS [19] and KAI1/CD82 [20]. And the previous studies have shown that these oncogenes can be taken as therapeutic targets to improve patient survival. The literature suggests that abnormal TRIM expression has a close association with the occurrence and progression of NSCLC. For example, highly expressed TRIM29 in NSCLC tissues indicates poor prognosis for NSCLC patients [21]. TRIM59 has a high expression level in a variety of lung cancer cell lines, while knockdown of which can affect the expression of cyclins (including CDC25C and CDK1), thereby enhancing the proliferative and migratory abilities of lung cancer cells [22]. TRIM44 displayed an upregulated expression in lung cancer cells, substantially facilitating invasion and migration of cancer cells [23]. However, the topic related to both TRIM66 and NSCLC is scarcely touched upon by researchers. In our study, q-PCR and Western blot pointed out that TRIM66 displayed a high expression level in NSCLC cells, which is consistent with the results of an existing study [24], which suggests that it may exert a promotive function in NSCLC.

Next, we knocked down TRIM66 expression to study its effect on the cellular phenotype of NSCLC and found that knocking down TRIM66 attenuated migration, invasion, and EMT process of cancer cells. Matrix metalloproteinases MMP2 and MMP9 are implicated in tumor angiogenesis and invasion [25], and these processes are regulated by some genes. For example, TGF-*β* mediates the regulation of MMP2 expression by exosome lnc-MMP2-2 to promote lung cancer cell invasion and migration [26]. EZH2 inhibits the transcription of TIMP2, which boosts activities of MMP-2 and MMP-9, which in turn increases the invasive activity of triple-negative breast cancer cells [27]. Therefore, influence of TRIM66 on migration and invasion of NSCLC cells may be realized by regulation of MMP2 or MMP9. Thus, we performed Co-IP to study the interaction between TRIM66 and MMP2 or MMP9 and found that there was a reciprocal relationship between TRIM66 and MMP9 only. Next, we found that silencing TRIM66 was capable of reversing promoting effect of MMP9 forced expression on migration, invasion, and EMT process of NSCLC cells by rescue experiment. Combined with the literature and our experimental results, TRIM66 promotes invasion, migration, and EMT in NSCLC by modulating MMP9.

Overall, we identified that both TRIM66 and MMP9 were upregulated in NSCLC cells. Silencing TRIM66 inhibits malignant progression of NSCLC cells, and this process is achieved by regulating MMP9. The findings may provide clues for elucidating the tumorigenesis of NSCLC and may offer a theoretical basis for generating novel approaches for NSCLC diagnosis and therapy.

The article "TRIM66 Promotes Malignant Progression of Non-Small-Cell Lung Cancer Cells via Targeting MMP9" was published in 2022. Journal: Comput Math Methods Med.

## Figures and Tables

**Figure 1:** TRIM66 is highly expressed in NSCLC cells. (a, b) Relative expression of TRIM66 mRNA and protein in human pulmonary alveolar epithelial and NSCLC cells; ^∗^*p* < 0.05.

**Figure 2:** TRIM66 knockdown inhibits the migration and invasion of NSCLC cells and EMT procession. (a, b) Expression levels of TRIM66 mRNA and protein in NSCLC cells after transfection with si-TRIM66. (c, d) Influence of knockdown of TRIM66 on cell migration and invasion. (e) Levels of EMT-related proteins; ^∗^*p* < 0.05.

**Figure 3:** The bindings between TRIM66 and MMP2 or MMP9. (a) Protein levels of MMP2 and MMP9 in each transfection group. (b) Cells were lysed and immunoprecipitated with antibodies, and immunocomplexes were analyzed by Western blot. (c) MMP9 level in proteins extracted from NSCLC and pulmonary alveolar epithelial cells.

**Figure 4:** TRIM66 affects progression of NSCLC cells by regulating MMP9. (a) Protein level of MMP9 in each group. (b, c) Migration and invasion of cells in each group. (d) Expression levels of EMT-related proteins; ^∗^*p* < 0.05.

**Table 1:** Information on antibodies used in the experiment.

Type	Name	Art. no.	Dilution rate
Primary antibodies (rabbit antibody)	TRIM66 polyclonal antibody	PA5-69788	1.0 *μ*g/mL
	MMP2 polyclonal antibody	PA5-85197	1 : 1000
	MMP9 polyclonal antibody	PA5-13199	1 : 2000
	E-cadherin polyclonal antibody	PA5-32178	1 : 1000
	N-cadherin polyclonal antibody	PA5-19486	1.0 *μ*g/mL
	Vimentin polyclonal antibody	PA5-27231	1 : 2000
	SNAIL polyclonal antibody	PA5-11923	1 : 1000
	*β*-Actin polyclonal antibody	PA5-16914	1.0 *μ*g/mL
Secondary antibody (goat anti-rabbit)	Goat anti-rabbit IgG H&L	A32731	0.1 *μ*g/mL

## Data Availability

The data used to support the findings of this study are available from the corresponding author upon request.

## References

[1] Bray F., Ferlay J., Soerjomataram I., Siegel R. L., Torre L. A., Jemal A. (2018). Global cancer statistics 2018: GLOBOCAN estimates of incidence and mortality worldwide for 36 cancers in 185 countries. *CA: a Cancer Journal for Clinicians*.

[2] Siegel R. L., Miller K. D., Jemal A. (2019). Cancer statistics, 2019. *CA: a Cancer Journal for Clinicians*.

[3] Ettinger D. S., Wood D. E., Aisner D. L. (2017). Non-small cell lung cancer, version 5.2017, NCCN clinical practice guidelines in oncology. *Journal of the National Comprehensive Cancer Network*.

[4] Evison M., AstraZeneca U. K. L. (2020). The current treatment landscape in the UK for stage III NSCLC. *British Journal of Cancer*.

The article "TRIM66 Promotes Malignant Progression of Non-Small-Cell Lung Cancer Cells via Targeting MMP9" was published in 2022. Journal: Comput Math Methods Med.

[5] Dai H. Y., Ma Y., Da Z., Hou X. M. (2018). Knockdown of TRIM66 inhibits malignant behavior and epithelial-mesenchymal transition in non-small cell lung cancer. *Pathology, Research and Practice*.

[6] Hatakeyama S. (2017). TRIM family proteins: roles in autophagy, immunity, and carcinogenesis. *Trends in Biochemical Sciences*.

[7] Ozato K., Shin D. M., Chang T. H., Morse H. C. (2008). TRIM family proteins and their emerging roles in innate immunity. *Nature Reviews. Immunology*.

[8] Ma Y., Dai H. Y., Zhang F., Zhao D. (2017). TRIM66 expression in non-small cell lung cancer: a new predictor of prognosis. *Cancer Biomarkers*.

[9] Nakashima H., Hashimoto N., Aoyama D. (2012). Involvement of the transcription factor twist in phenotype alteration through epithelial-mesenchymal transition in lung cancer cells. *Molecular Carcinogenesis*.

[10] Thomson S., Petti F., Sujka-Kwok I. (2011). A systems view of epithelial-mesenchymal transition signaling states. *Clinical & Experimental Metastasis*.

[11] He T., Cui J., Wu Y., Sun X., Chen N. (2019). Knockdown of TRIM66 inhibits cell proliferation, migration and invasion in colorectal cancer through JAK2/STAT3 pathway. *Life Sciences*.

[12] Huang H. (2018). Matrix metalloproteinase-9 (MMP-9) as a cancer biomarker and MMP-9 biosensors: recent advances. *Sensors*.

[13] Xue Q., Cao L., Chen X. Y. (2017). High expression of MMP9 in glioma affects cell proliferation and is associated with patient survival rates. *Oncology Letters*.

[14] Chen S. W., Zhang Q., Xu Z. F. (2016). HOXC6 promotes gastric cancer cell invasion by upregulating the expression of MMP9. *Molecular Medicine Reports*.

[15] Tripathy J., Tripathy A., Thangaraju M., Suar M., Elangovan S. (2018). *α*-Lipoic acid inhibits the migration and invasion of breast cancer cells through inhibition of TGF*β* signaling. *Life Sciences*.

[16] Zhang H., Hao C., Wang Y. (2016). Sohlh2 inhibits human ovarian cancer cell invasion and metastasis by transcriptional inactivation of MMP9. *Molecular Carcinogenesis*.

[17] Dong H., Diao H., Zhao Y. (2019). Overexpression of matrix metalloproteinase-9 in breast cancer cell lines remarkably increases the cell malignancy largely via activation of transforming growth factor beta/SMAD signalling. *Cell Proliferation*.

[18] Shay G., Lynch C. C., Fingleton B. (2015). Moving targets: emerging roles for MMPs in cancer progression and metastasis. *Matrix Biology*.

[19] Román M., Baraibar I., López I. (2018). KRAS oncogene in non-small cell lung cancer: clinical perspectives on the treatment of an old target. *Molecular Cancer*.

[20] Prabhu V. V., Devaraj S. N. (2017). KAI1/CD82, metastasis suppressor gene as a therapeutic target for non-small-cell lung carcinoma. *Journal of Environmental Pathology, Toxicology and Oncology*.

The article "TRIM66 Promotes Malignant Progression of Non-Small-Cell Lung Cancer Cells via Targeting MMP9" was published in 2022. Journal: Comput Math Methods Med.

[21] Song X., Fu C., Yang X., Sun D., Zhang X., Zhang J. (2015). Tripartite motif-containing 29 as a novel biomarker in non-small cell lung cancer. *Oncology Letters*.

[22] Zhan W., Han T., Zhang C. (2015). TRIM59 promotes the proliferation and migration of non-small cell lung cancer cells by upregulating cell cycle related proteins. *PLoS One*.

[23] Luo Q., Lin H., Ye X., Huang J., Lu S., Xu L. (2015). Trim44 facilitates the migration and invasion of human lung cancer cells via the NF-*κ*B signaling pathway. *International Journal of Clinical Oncology*.

[24] Zhang Y., Wu L., Jiang C., Yan B. (2015). Reprogramming cellular signaling machinery using surface-modified carbon nanotubes. *Chemical Research in Toxicology*.

[25] Farina P., Tabouret E., Lehmann P. (2017). Relationship between magnetic resonance imaging characteristics and plasmatic levels of MMP2 and MMP9 in patients with recurrent high-grade gliomas treated by bevacizumab and irinotecan. *Journal of Neuro-Oncology*.

[26] Wu D. M., Deng S. H., Liu T., Han R., Zhang T., Xu Y. (2018). TGF-*β*-mediated exosomal lnc-MMP2-2 regulates migration and invasion of lung cancer cells to the vasculature by promoting MMP2 expression. *Cancer Medicine*.

[27] Chien Y. C., Liu L. C., Ye H. Y., Wu J. Y., Yu Y. L. (2018). EZH2 promotes migration and invasion of triple-negative breast cancer cells via regulating TIMP2-MMP-2/-9 pathway. *American Journal of Cancer Research*.

